RETRACTED

# Feasibility of Constructing an Automatic Meniscus Injury Detection Model Based on Dual-Mode Magnetic Resonance Imaging (MRI) Radiomics of the Knee Joint

**DOI:** 10.1155/2022/2155132

**Published:** 2022-03-29

**Authors:** Yi Wang, Yuanzhe Li, Meiling Huang, Qingquan Lai, Jing Huang, Jiayang Chen

**Affiliations:** ^1^Department of CT/MRI, The Second Affiliated Hospital of Fujian Medical University, Quanzhou 362000, China; ^2^Radiology Department, The Second Affiliated Hospital of Fujian Medical University, Quanzhou 362000, China; ^3^Radiology Department, Anxi Hospital of Traditional Chinese Medicine, Quanzhou 362400, China

## Abstract

**Objective:**

To explore the feasibility of automatically detecting the degree of meniscus injury by radiomics fusion of dual-mode magnetic resonance imaging (MRI) features of sagittal and coronal planes of the knee joint.

**Methods:**

This retrospective study included 164 arthroscopically confirmed meniscus injuries in 152 patients admitted to the Department of Orthopaedics of our hospital from July 2018 to March 2021. A total of 1316-dimensional radiomics signatures were extracted from single-mode sagittal and coronal plane images of menisci, respectively. Then, the sagittal and coronal plane features were fused to form a dual-mode joint feature group with a total of 2632-dimensional radiomics signatures. The minimum redundancy maximum relevance (mRMR) algorithm and the least absolute shrinkage and selection operator (LASSO) regression were used to select features and generate optimal radiomics signatures. The single-mode sagittal plane feature model (Model 1), single-mode coronal plane feature model (Model 2), and the combined sagittal and coronal plane feature model (Model 3) performance were tested by receiver operating characteristic (ROC) curves and Delong test. The calibration curve test was used to verify the reliability of radiomics signatures of the three models.

**Results:**

The average intra- and interobserver intraclass correlation coefficients (ICCs) of the most significant 8-dimensional radiomics signatures of Model 1 and Model 2 were 0.935 (range 0.832-0.998) and 0.928 (range 0.845-0.998), respectively. All the three models had good detection performance; Model 3 had the most significant performance (the areas under the curve (AUCs) of training, and validation sets were 0.947 and 0.923, respectively), which was superior to Model 1 (AUCs of training set and validation set were 0.889 and 0.876, respectively) and Model 2 (AUCs of training set and validation set were 0.831 and 0.851, respectively). The detection probability of training and validation sets in the three models was highly consistent with the actual clinical probability.

RETRACTED

**Conclusions:**

It is feasible to establish a model for automatic detection of meniscus damage by means of radiomics. The detection performance of the dual-mode knee MRI model is better than that of any single-mode model, showing potent feature analysis ability and outstanding detection performance.

## 1. Introduction

Meniscus injury is the most common type of knee injury, which can be divided into meniscus tear and meniscus degeneration [1, 2]. The treatment of meniscus injury varies, depending on the degree of injury. Therefore, the degree of meniscus injury must be determined first before formulating a scientific treatment plan for targeted treatment. In clinical practice, arthroscopy is considered the gold standard for diagnosing meniscus injury, with an accuracy rate of 98.6%. However, due to the traumatic nature of arthroscopy, a noninvasive and accurate inspection method is needed to accomplish this task. Currently, magnetic resonance imaging (MRI) is recognized as a detection method with high accuracy [3, 4], with the accuracy rate reaching 85%-90% under favorable conditions [5, 6], whereas judging the degree of meniscus injury depends more on the radiologist's working experience and the interpretation of a large amount of image data.

At present, the medical image data shows an explosive growth with a lot of interference and useless information, which virtually brings a challenge to the professional ability of doctors and restricts the accuracy of judgment. Therefore, it is particularly important to carry out efficient, accurate, and effective information mining. Radiomics, an effective method for extracting key parameters from medical images, is also a powerful tool to guide diagnosis and treatment in modern medicine. In recent years, it has been applied in many fields such as the research on tumor diagnosis and treatment [7–9], mental diseases, and heart diseases [10, 11], with encouraging results. But studies on meniscus injuries are relatively rare and recent.

In known studies, researchers used the deep approach of learning to extract features from MRI images of knee joints and detect injuries [12, 13] and found that this method was feasible to detect meniscus injuries [12, 14]. In other disease areas, Abd-Ellah et al. [15] proved the superiority of the proposed deep learning-based method for tumor detection and demonstrated the advantage of the whole system's performance concerning both tumor detection and localization measures. In addition, Bien et al. [16] developed a deep learning model that achieves high performance in clinical classification tasks on knee MRI and demonstrated the benefits, in a retrospective experiment, of providing model predictions to clinicians during the diagnostic imaging task. Although some progress has been made in the detection of meniscus injury by deep approach of learning, most of the studies focus on the binary-class classification of detecting meniscus injury (with or without), and there is little research on distinguishing meniscus degeneration from meniscus tear. Moreover, the deep approach of learning is subject to the influence of existing technologies, research methods, datasets, etc., so it still goes a long way before extensive promotion.

RETRACTED

Therefore, the novelty and motivation of the study is to distinguish meniscus degeneration from meniscus tear and automatically detect different degrees of meniscus injury by fusing the features of MRI images of sagittal and coronal planes of the knee joint, which is rarely reported both at home and abroad. It is hoped that a model for automatic detection of meniscus damage can be established by means of radiomics.

## 2. Materials and Methods

### 2.1. Source of Cases

The ethical approval of this retrospective study was provided by the Ethics Review Committee of our hospital, with the Ethics No. of [2021] No. 303 of the second Affiliated Hospital of Fujian Medical University. All patient information was kept strictly confidential. A total of 164 injured meniscals (per side) were collected from 152 patients admitted to the Department of Orthopaedics of the second Affiliated Hospital of Fujian Medical University from July 2018 to March 2021. All patients had arthroscopically confirmed meniscus injury and underwent MRI of the affected knee. Among the 152 patients, 97 were males and 55 were females, ranging in age from 9 to 76 years old, with an average of 52.4 ± 11.0 years. Meniscus injury was divided into meniscus tear and meniscus degeneration. Among the 164 meniscus injuries, 78 meniscus tears and 86 meniscus degeneration were found. The results of arthroscopy were obtained by orthopedic specialists with rich experience in arthroscopic surgery. MRI images of all menisci in enrolled patients were randomly divided into a training set and a validation set (7 : 3). The same proportion of meniscus degeneration and meniscus tear were maintained in the training and validation sets using stratified random sampling. The flow chart of the study is shown in Figure 1.

Inclusion criteria were as follows: patients with arthroscopically confirmed meniscus injury and patients who underwent MRI scanning before treatment.

Exclusion criteria were as follows: treatment before MRI scanning; unavailable or incomplete clinical or MRI information; poor MRI image quality with low signal-to-noise ratio (SNR); pregnant women and lactating patients; patients with metal implants; and patients with claustrophobia or other inability to cooperate with the examination.

RETRACTED

### 2.2. MRI Image Acquisition and Arthroscopic Acquisition

All patients were examined by the Philips 3.0 T MRI system (Achieva, Philips Healthcare, Best, the Netherlands), which was equipped with a dedicated 15-channel transmitting/receiving knee joint coil. Fixed with a sandbag on the lower leg, the patient was instructed to maintain the static orientation of the knee during the scan on the coronal and sagittal planes. The scanning center was horizontal to the articular space, the coronal scanning line was parallel to the tibial plateau, and the sagittal scanning line was perpendicular to the tibial plateau. The scanning parameters are as follows: T1WITR spin echo (SE) sequence = 450-500 ms, TE = 14 ms, average number of times = 2; gradient echo (MED) sequence T2 WI TR = 800-1000 ms, TE = 26 ms, matrix = 256 × 256, average number of times = 1, and flip angle = 30°. The layer spacing and thickness were 1 mm and 3 mm, respectively. Arthroscopy: The operating system of arthroscopy was digitalized by STRYKER, USA.

### 2.3. Segmentation of Region of Interests (ROIs)

All ROIs were completed independently by a radiologist (reader A, a radiologist with 10 years of musculoskeletal experience and no knowledge of the final diagnosis) using ITK-SNAP 3.6.0, and meniscus images were manually segmented along each sagittal and coronal section of the ipsilateral meniscus (Figure 2). Referring to the previous radiomics study that required segmentation [17, 18], all lesions were resegmented by reader A one month later to evaluate the intraobserver consistency of the two segmentations. All lesions were redivided independently by another senior radiologist (reader B, a radiologist with 15 years of musculoskeletal experience and no knowledge of the final diagnosis) to assess the interobserver consistency. Intra- and interobserver intraclass correlation coefficients (ICCs) were used to determine the consistency of feature extraction. Any ICC greater than 0.80 was classified as good consistency.

### 2.4. Extraction, Screening, and Modeling of Radiomics Signatures

Using the radiomics module inserted in the AK software (artificial intelligence toolkit; GE Healthcare), 1316-dimensional radiomics signatures were extracted from the single-mode sagittal and coronal planes of menisci, respectively. Then, the sagittal and coronal plane features were fused to form a dual-mode joint feature group with a total of 2632-dimensional radiomics signatures. All the extracted features can be subdivided into the following categories: first-order statistics, shape-based, gray-level cooccurrence matrix (GLCM), gray-level size zone matrix (GLSZM), gray-level run-length matrix (GLRLM), first-order function (FIRSTORDER), and gray-level difference matrix (GLDM). A detailed description of the radiomics signatures can be found on the PyRadiomics Documentation website (http://pyradiomics. readthedocs.io).

RETRACTED

The obtained features were normalized, and the unit limit was removed. For highly reproducible image features (intraobserver and interobserver ICCs >0.80), the minimum redundancy maximum relevance (mRMR) algorithm [19] is helpful to eliminate confounding factors. The extracted features were then indexed according to their correlation redundancy index. mRMR and the least absolute shrinkage and selection operator (LASSO) [20], both of which are feature selection methods, were used to select the most useful features in the training set. First, the mRMR algorithm, a multivariable ranking method, was used to rank features according to the correlation redundancy index of features based on heuristic evaluation criteria, and the top 20 features with the highest correlation were selected. Then, LASSO regression was performed using 10-fold cross-validation on the training set. The optimized feature subset was selected to further construct radiomics signatures, and the corresponding coefficients were calculated. Radiomics signatures were obtained by adding the selected texture features and weighting them by their respective coefficients. Then, the optimal feature subset was selected by the LASSO method to build the final model. The function of LASSO algorithm includes selecting regularization parameters and determining the number of selected features. Finally, an automatic detection model of meniscus injury degree was established by LASSO regression based on the selected radiomics signatures. In this study, the model established by sagittal plane images was defined as Model 1, the model established by coronal plane images was defined as Model 2, and the combined model of sagittal and coronal plane images was defined as Model 3. The whole process of data collection, lesion segmentation, feature extraction, feature selection, and model building in this study is shown in the flow chart.

### 2.5. Statistical Analysis

This study used SPSS 24.0 (SPSS, Inc., Chicago, IL, USA) software and R software (version 3.5.0; http://www.R-project.org/) for statistical analysis. Receiver operating characteristic (ROC) curves were drawn to determine the detection performance of the three models. Then, the area under the curve (AUC), as well as sensitivity, specificity, and accuracy were determined by the Youden index. The Delong test was performed for pairwise comparison of the detection performance among the three models. The detection probability of Model 3 was analyzed by Logistic regression. Calibration curves were used to determine the reliability of image features of the three models.

RETRACTED

## 3. Results

### 3.1. Construction of Radiomics Signatures

Among the 1316-dimensional radiomics signatures of the single-mode model, 981 with intraobserver and interobserver ICCs >0.80 were retained. The mRMR algorithm eliminated 981-dimensional radiomics signatures and retained 20-dimensional features (Figure 3). The optimal subset of features selected by LASSO regression and the determined features are shown in Figure 4. In the training set, the most significant 8-dimensional features of Model 1 and Model 2 were selected (Figures 4(a) and 4(b)), and the radiomics signatures were established by LASSO regression. The average intra- and interobserver ICCs of the most significant 8-dimensional radiomics signatures of Model 1 and Model 2 were 0.935 (range 0.832-0.998) and 0.928 (range 0.845-0.998), respectively (Table 1). Among the 2632-dimensional radiomics features of the dual-mode model, 1962 with intragroup and intergroup ICCs >0.80 were retained. After preserving 20-dimensional features using the mRMR algorithm (Figures 3(e)–3(f)), 9-dimensional features with the greatest contribution were retained by LASSO regression, including single-mode sagittal and coronal plane features, among which 6 sagittal plane features and 3 coronal plane features were extracted (Figure 4(c)). The feature map was sorted by the importance of features, and the ordinate was the coefficient. The larger the coefficient, the more obvious the contribution rate of the feature.

### 3.2. Performance of Radiomics Models

This study examined the performance of the three models (Figure 5). In Model 1, the AUC value, accuracy, sensitivity, and specificity of radiomics signatures in the training set were 0.889, 0.873, 0.869, and 0.881, respectively (95% confidence interval [CI]: 0.845-0.942, *P* < 0.001, Figure 5(a)). The AUC value of radiomics signatures in the validation set was 0.876, and the accuracy, sensitivity, and specificity were 0.862, 0.871, and 0.855, respectively (95% CI 0.875-0.984, *P* < 0.001, Figure 5(d)). In Model 2, the AUC value of radiomics signatures in the training set was 0.831, and the accuracy, sensitivity, and specificity were 0.836, 0.878, and 0.846, respectively (95% CI: 0.875-0.984, *P* < 0.001, Figure 5(b)); the AUC, accuracy, sensitivity, and specificity of radiomics signatures in the validation set were 0.851, 0.879, 0.847, and 0.853, respectively (95% CI: 0.834-0.921, *P* < 0.001, Figure 5(e)). In Model 3, the AUC value of radiomics signatures in the training set was 0.947, and the accuracy, sensitivity, and specificity were 0.863, 0.874, and 0.886, respectively (95% CI: 0.865-0.944, *P* < 0.001, Figure 5(c)); The AUC, accuracy, sensitivity, and specificity of radiomics signatures in the validation set were 0.923, 0.891, 0.889, and 0.895, respectively (95% CI: 0.829-0.996, *P* < 0.001; Table 2, Figure 5(f)).

RETRACTED

Verification was performed on the training set and the validation set of the three models using the calibration curves, and the results showed that the detection probability of both sets in the three models was highly consistent with the actual clinical probability (Figure 6). Pairwise comparisons of the three ROC curves (Model 1, Model 2, and Model 3) were performed by the Delong test, and the results showed that (Table 3) the *P* value of the ROC curve of Model 1 and Model 2 was 0.0447, suggesting that the detection performance of the sagittal model was significantly better than that of the coronal model; the *P* value of the ROC curve of Model 3 and Model 1 was 0.0216, which indicated that the performance of the dual-mode model was significantly better than that of the sagittal model; the *P* value of the ROC curve of Model 3 and Model 2 was 0.0309, suggesting that the performance of the dual-mode model was significantly better than that of the coronal model.

## 4. Discussion

Meniscus injury, a common type of knee joint injury, will easily lead to a series of clinical diseases such as knee joint pain and osteoarthritis without proper treatment [21, 22]. Correct judgment of meniscus injury degree is an important prerequisite for clinical intervention. At present, radiomics-based disease detection is a brand new field that has been applied to perform a wide range of radiological tasks. We believe that it is suitable to model the complex relationship between medical images and diagnosis by extracting high-throughput texture features from images. The advantage lies in extracting information from large-scale images of imaging systems to the maximum extent, filtering a large amount of interference information in images, and improving image interpretation by reducing the human error rate. Based on previous research of radiomics in other diseases [7–9], we found that the new data could be classified by using LASSO regression as a stable variable filter and combining the radiomics signatures with LASSO regression to construct a model through automatic learning, extraction, and screening of MRI images of menisci. By transforming the sectional image array into quantifiable features, a model with strong detection ability is established. Therefore, this study attempts to use radiomics to help quickly detect the extent of meniscus injury to guide further treatment.

RETRACTED

Recently, the feasibility of artificial intelligence-based meniscus tear detection on MRI images has been confirmed [1, 2, 23, 24]. However, to date, there are few artificial intelligence training software algorithms that can successfully and comprehensively evaluate the complete cross-sectional imaging research in musculoskeletal radiology. In addition, these studies mainly focused on automatic meniscus segmentation and tear detection by the deep approach of learning. Although the detection performance is improving year by year, its ability to be generalized is limited by the fact that sufficient training usually requires processing large amounts of data and requires huge computing power.

In this study, we used radiomics signatures based on MRI of the knee joint to distinguish meniscus degeneration from meniscus tear. ROC analysis revealed high performance of the radiomics model. The results showed that in the training set and validation set of Model 1, Model 2, and Model 3, the AUCs of the radiomics signatures were 0.889 and 0.876, 0.831 and 0.851, and 0.947 and 0.923, respectively, indicating that there were significant differences in heterogeneity between meniscus degeneration and meniscus tear. Hence, the selected radiomics signatures may be able to detect the difference between the two. In addition, the results showed that the detection models used to distinguish meniscus degeneration and meniscus tear had good performance, which was higher than the results of Bien et al. [16] in 2018, and similar to the results of Fritz and Astuto et al. in predicting the severity of meniscus injury [25, 26]. The results of the Delong test revealed that the sagittal model was superior to the coronal model and the dual-mode radiomics model was superior to any cross-sectional model. Further, calibration curves were plotted to verify the reliability of the three models, and the results showed that the detection ability of the three models was infinitely close to the actual clinical results. According to the above results, we believe that it is feasible to construct an automatic meniscus injury detection model using the radiomics method and that the radiomics method has a good ability to automatically distinguish meniscus degeneration from meniscus tear.

In clinical practice, we often have to face interference factors that affect the accurate judgment of meniscus injury. For example, in some cases, structures such as the ligaments of Humphry and Wrisberg are mistaken as the damaged part. Moreover, partial truncation artifact and magic angle effect can cause signals similar to mild tear at the edge of the meniscal body [27]. All these factors seriously restrict radiologists to accurately assess the degree of meniscus injury. In this study, LASSO classifier was used to classify meniscus degeneration and meniscus tear, and the optimal features were extracted from the three models to quantify meniscus MRI images. LASSO regression can select more meaningful independent variables by compressing the coefficients of some meaningless or insignificant independent variables to zero. By analyzing these features, we found that changes in MRI signals and the extent of meniscus injury were important factors in distinguishing degenerative changes from tears, which was in agreement with the traditional MRI diagnosis of meniscus injury. Through the features extracted from Model 3, we found that the dual-mode radiomics model could fuse several optimal image features of both the sagittal and coronal planes, comprehensively covering several major features of the injury. Moreover, the number and coefficients of sagittal features were higher than those of coronal features, which demonstrated that sagittal plane radiomics signatures were superior to coronal plane features.

RETRACTED

In this study, a dual-mode radiomics model was used to comprehensively analyze the MRI image feature differences between different degrees of meniscus injury, which is helpful for radiologists to deepen their understanding of the characteristics of meniscus injury, reduce the influence of some interference factors on the accurate diagnosis of different degrees of meniscus injury, and prevent unnecessary trauma caused by arthroscopic overexamination, especially when meniscus degeneration is suspected, so as to achieve the purpose of improving the detection efficiency of radiologists and orthopedic surgeons and saving medical resources.

While the findings in this paper provide promising insights, there are some limitations. First of all, as a small-scale study, sample size is a problem. Second, all ROIs in this study were manually segmented, which is an intensive and time-consuming process without any automatic segmentation algorithm. Manual segmentation still has a long way to go to match the accuracy and reproducibility of automatic segmentation. Efficient segmentation algorithms for ROIs are needed to be studied. Finally, although the radiomics processing flow of this study has been relatively perfected, there are still some deficiencies, which need to be continuously improved and optimized in future research. Radiomics can be used as a complement to other omics such as proteomics and genomics. Therefore, it is worth expecting that the combination of multiple omics will be the best choice for the treatment of diseases. With the in-depth development of radiomics research, we will increase the number of research samples and optimize the operation process on the basis of this research to achieve further improvement.

RETRACTED

## 5. Conclusion

This study finds that it is feasible to establish an automatic detection model for different degrees of meniscus injury by means of radiomics. The detection performance of the dual-mode knee joint MRI radiomics model is better than that of any single-mode model, showing strong feature analysis ability and outstanding detection performance. It is hoped that in future research, the radiomics method can provide more rapid and effective help for radiologists and orthopedic surgeons.

## Figures and Tables

**Figure 1:** Flow chart.

**Figure 2:** Dual-mode MRI of the knee joint ((a) tear of the posterior horn of the medial meniscus of the right knee joint; (b) degeneration of the medial meniscus of the right knee joint; the red area is the manually segmented meniscus image).

**Figure 3:** LASSO regression is performed based on the regularization parameter (*λ*) to determine the number of features ((a) cross-validated MSE of LASSO fit in Model 1; (b) trace plot of coefficients fit by LASSO in Model 1; (c) cross-validated MSE of LASSO fit in Model 2; (d) trace plot of coefficients fit by LASSO in Model 2; (e) cross-validated MSE of LASSO fit in Model 3; (f) trace plot of coefficients fit by elastic net in Model 3).

**Figure 4:** The most predictive subset of features and the corresponding coefficients ((a) 8 optimal sagittal features extracted in Model 1; (b) 8 optimal coronal features extracted in Model 2; (c) 9 optimal features of the combined sagittal and coronal planes extracted in Model 3).

**Figure 5:** Performance evaluation curve of MRI automatic detection model for meniscus injury degree ((a) ROC curves of the training set of Model 1; (b) ROC curves of the training set of Model 2; (c) ROC curves of the training set of Model 3; (d) ROC curves of the validation set of Model 1; (e) ROC curves of the validation set of Model 2; (f) ROC curves of the validation set of Model 3).

**Figure 6:** Calibration curves are used to verify the reliability of the training and validation sets of models ((a) training set of Model 1; (b) validation set of Model 1; (c) training set of Model 2; (d) validation set of Model 2; (e) training set of Model 3; (f) validation set of Model 3).

**Table 1:** ICCs of the remaining eight features after Model 1 and Model 2 redundancy analysis.

Groups	Radiomics signatures	Intraobserver ICCs	Interobserver ICCs
Model 1	logsigma50mm3D_glcm_InverseVariance_sag	0.994	0.982
	square_glszm_ZoneEntropy_sag	0.995	0.998
	logsigma50mm3D_glcm_Correlation_sag	0.983	0.916
	logsigma50mm3D_firstorder_Skewness_sag	0.832	0.814
	logarithm_gldm_LargeDependenceEmphasis_sag	0.891	0.923
	logarithm_glcm_DifferenceAverage_sag	0.962	0.971
	logsigma40mm3D_glszm_SmallAreaEmphasis_sag	0.891	0.845
	original_gldm_LowGrayLevelEmphasis_sag	0.990	0.911

Model 2	square_glcm_Imc2_cor	0.936	0.901
	waveletHHH_gldm_LowGrayLevelEmphasis_cor	0.877	0.921
	logsigma50mm3D_glcm_InverseVariance_cor	0.964	0.991
	waveletHHH_gldm_LargeDependenceLowGrayLevelEmphasis_cor	0.881	0.934
	logsigma50mm3D_firstorder_Maximum_cor	0.827	0.869
	waveletLLL_firstorder_Kurtosis_cor	0.937	0.892
	waveletHHH_glrlm_ShortRunEmphasis_cor	0.998	0.987
	logsigma50mm3D_glcm_Idmn_cor	0.995	0.998

RETRACTED

**Table 2:** The area under the ROC curve (AUC), accuracy, sensitivity, and specificity of training set and validation set of Model 1, Model 2, and Model 3.

Groups	AUC	Accuracy	Sensibility	Specificity	95% confidence interval
Model 1					
Training set	0.889	0.873	0.869	0.881	0.845-0.942
Validation set	0.876	0.862	0.871	0.855	0.875-0.984
Model 2					
Training set	0.831	0.836	0.878	0.846	0.875-0.984
Validation set	0.851	0.879	0.847	0.853	0.834-0.921
Model 3					
Training set	0.947	0.863	0.874	0.886	0.865-0.944
Validation set	0.923	0.891	0.889	0.895	0.829-0.996

**Table 3:** Delong test on the ROC curves of Model 1, Model 2, and Model 3 for detection efficiency.

Grouping	*P* value
Model 1 and Model 2	0.045
Model 3 and Model 1	0.022
Model 3 and Model 2	0.031

## Data Availability

The labeled dataset used to support the findings of this study are available from the corresponding author upon request.
